# Evaluation of Short-Term Insulin Pump for Treatment of Patients with Type 2 Diabetes Mellitus Complicated with Lower Extremity Arterial Disease in Endocrinology by Ultrasonography

**DOI:** 10.1155/2022/9128208

**Published:** 2022-05-27

**Authors:** Qiongyao Guo, Zhouyue Li, Hua Chen

**Affiliations:** ^1^Department of Endocrinology, The People's Hospital of Putuo Zhoushan, Zhoushan, 316100 Zhejiang, China; ^2^Department of Ultrasound, The People's Hospital of Putuo Zhoushan, Zhoushan, 316100 Zhejiang, China

## Abstract

This research aimed to explore the curative effect of short-term insulin pump in the treatment of type 2 diabetes mellitus (T2DM) patients with lower extremity arterial disease (LEAD) based on ultrasonography. 422 patients (220 males and 202 females) with T2DM in the hospital were selected, and they were randomly divided into control group (*n* = 211, oral hypoglycemic drugs or diet control, appropriate exercise to lower blood glucose) and experimental group (*n* = 211, insulin pump was used to reduce blood glucose). After 2 weeks, the therapeutic effect was evaluated by ultrasonography. The results showed that after two weeks of treatment, the difference in lumen intima between the two groups was statistically significant (*P* < 0.05). The intima-media thickness (IMT) values of the experimental group were 0.83 ± 0.03 mm, 0.62 ± 0.03 mm, and 0.41 ± 0.04 mm, respectively, which were significantly different from those of the control group (1.62 ± 0.54 mm, 1.23 ± 0.14 mm, and 0.78 ± 0.11 mm) (*P* < 0.05). There was obvious difference in low-density lipoprotein cholesterol (LDL-C) level between the experimental group (2.22 ± 0.46 mmol/L) and the control group (3.21 ± 0.62 mmol/L) (*P* < 0.05). The LEAD score of the experimental group was 5.51 ± 1.11, which was significantly different from that of the control group (7.08 ± 2.73) (*P* < 0.05). There was clear difference in LEAD score between the two groups under different course of disease (CD) (*P* < 0.05). Studies indicated that short-term application of insulin pump therapy could effectively improve the pathological changes of lower limbs in patients with T2DM, which had clinical application value.

## 1. Introduction

In recent years, the incidence of diabetes mellitus (DM) has increased year by year [1]. The blood glucose concentration in patients with DM is high, and long time in this state will affect the metabolic function of the body [2]. Especially in patients with large changes in blood glucose concentration and poor control, which is often prone to concurrent infectious diseases, the symptoms are generally more serious, and it is difficult to control [3]. Among the chronic complications, vascular lesions have the highest prevalence [4]. Diabetic microangiopathy mainly includes diabetic retinopathy and diabetic nephropathy, and cerebral artery, aorta, coronary artery, and limb artery are the more common arteries in diabetic macroangiopathy [5].

Diabetic lower extremity arterial disease (LEAD) is a manifestation of diabetic macrovascular complications in the lower extremities. High blood glucose concentration will directly affect the intima. In addition to the combined action of various types of inflammatory cells, it eventually causes lower extremity atherosclerosis. After vulnerable plaque detachment, it causes that the blood cannot circulate normally in the peripheral arteries, or secondary ulcer and bleeding, resulting in the formation of thrombosis. If the disease continues to develop, the diameter of the vessel becomes smaller or even occluded, resulting in reduced or even no blood supply to the peripheral blood of the limbs, and blood circulation disorders are caused [6]. The most typical clinical symptom of LEAD is intermittent claudication, but because patients with type 2 diabetes mellitus (T2DM) are complicated by peripheral neuropathy, they generally do not experience significant clinical symptoms. Patients' leg symptoms are often atypical or even have no special manifestations, they generally go to the hospital when gangrene, tissue necrosis, and severe resting pain occur, and the diseases often have progressed to the stage of critical limb ischemia when diagnosed [7]. LEAD can not only lead to gangrene or even amputation but also increase the risk of cardiovascular events and mortality in patients [8]. Early diagnosis of LEAD and delaying its appearance and development are of great value in reducing the burden on patients and improving patients' quality of life.

DSA is currently the gold standard for the diagnosis of vascular diseases in clinical practice, which can clearly show where embolism or stenosis occurs in the lower extremity vessels, as well as the location, shape, and size of abnormal plaques. However, DSA examination is an invasive examination, which will have a certain impact on the patient's body, such as radiation; in addition, the use of contrast agent will also have a certain toxicity to the heart and kidney, and its required cost is high, so it cannot be the preferred method for clinical examination [9]. CTA is a method that can quickly and clearly show the vascular structure, the location of the lesion, the extent of lesion involvement, and the anatomical relationship between the diseased vessel and the surrounding tissues; however, its diagnostic ability will be affected by calcification; moreover, CTA cannot dynamically show arterial filling, and is susceptible to artifacts interference for small vessel display [10]. MRA is a vascular detection method emerging with the development of magnetic resonance imaging technology. Clinically, through the use of contrast agent, the signals between blood vessels and surrounding tissues will form significant differences, which can more prominently show vascular lesions. However, MRA image acquisition is time-consuming and relatively expensive, and if a metal foreign body remains in the patient, the patient cannot undergo MRA examination [11]. Ultrasonography plays an irreplaceable role in the imaging examination of vascular lesions. It is characterized by noninvasive, short time-consuming, real-time, inexpensive, and repeatable comparison and tracking. Numerous studies have shown that ultrasonography has a high diagnostic efficacy for varying degrees of stenosis and occlusion of lower extremity arteries and a high diagnostic value for LEAD [12].

Since the destruction of islet function by poor control of blood glucose in the early stage can be reversed, if new-onset T2DM can be enhanced as early as possible, supplemented by standardized diet and exercise therapy to restore blood glucose to nearly normal levels, it can maximize the improvement of injured islet function and even enable some patients to obtain long-term remission through the improvement of early metabolic memory effect [13]. As an effective and stable hypoglycemic means, insulin pump therapy reduces the adverse reactions caused by the increase in the dosage of oral drugs and enhances the compliance of patients. It is generally more suitable for patients with T2DM who have severely elevated blood glucose needed to be rapidly controlled [14]. If the body is in a hyperglycemic environment for a long time, the risk of various related complications such as retinopathy, neurological, and renal system diseases in the future will be significantly increased compared with those treated early.

Therefore, patients with T2DM and LEAD were selected and treated with insulin pump, which was compared with oral hypoglycemic drugs, and ultrasound images were applied to assess the patient's lower limb vascular status after treatment to explore its short-term therapeutic effect. It provides reference value for the treatment of T2DM patients with LEAD in clinical practice to improve the therapeutic effect.

## 2. Research Methods

### 2.1. Research Subjects

A total of 422 diagnosed T2DM patients with LEAD (220 males and 202 females) in hospital from June 2017 to June 2020 were selected. The patients were randomly divided into control group (*n* = 211): close monitoring of blood glucose, oral hypoglycemic drugs or diet control, and appropriate exercise to lower blood glucose; and experimental group (*n* = 211): insulin pump was used for about 2 weeks to reduce blood glucose according to the treatment methods used in the initial diagnosis of medical records. In the control group, the mean age was 45.42 ± 4.12 years, the mean course of disease (CD) was 10.11 ± 6.52 years, and the mean BMI level was 24.18 ± 1.34 kg/m^2^; in the experimental group, the mean age was 46.25 ± 3.28 years, the mean CD was 11.32 ± 5.39 years, and the mean BMI level was 24.93 ± 1.19 kg/m^2^. The study had been approved by the ethics committee of the hospital. The patients and their families signed the informed consents.

The diagnosis and classification of patients referred to the relevant guidelines published by WHO in 1999: all subjects had a minimum fasting time of 10 hours, the elbow vein was selected for blood sampling, 75 g of glucose was dissolved in 300 mL of warm boiled water, so that the subjects took it at one time (within 5 minutes). Blood samples were taken through the vein 1 hour and 2 hours later, respectively, and the samples taken twice were determined.

Inclusion criteria: patients with DM symptoms and blood glucose ≥ 11.1 mol/L at any time after meal; FPG ≥ 7.0 mmol/L patients; patients with 2hPG ≥ 11.1 mmol/L in OGTT trial. Exclusion criteria: T1DM patients; those in pregnancy or lactation; patients with acute and chronic infection, traumatic surgery, and other stress events: patients with acute metabolic disorders; patients suffering from serious cardiovascular and cerebrovascular diseases; patients with diseases that are not cured and have an impact on prognosis: patients with active or inactive malignant tumors, psychiatric, blood, and skin diseases; patients who may cause diseases related to abnormal glucose metabolism or need drugs that may cause disorders of glucose metabolism: patients with thyroid diseases and immune-related diseases.

### 2.2. Insulin Pump Therapy

Patients and their families were given diabetes education, and patients were given appropriate nutritional therapy and assistance in the development of individualized DM recipes and reasonable exercise plans. Before treatment, insulin pump working principle was informed, and after fasting for ≥10 h, venous blood was taken by nursing staff for FPG, lipid profile, liver and kidney function, HbA1c, and HCY detection in the next morning. After blood collection, the patients in the experimental group received intensive insulin pump therapy for 2 weeks. During this period, the blood glucose was measured by a specially-assigned person before and after three meals, before bedtime, and at 3 : 00 am daily. When the FPG and PPG of the patients under 70 years old were close to normal, it was considered that the blood glucose control was up to standard; when the FPG of the patients over 70 years old was 6-8 mmol/L, 2 h PG 8-10 mmol/L, it was considered that the blood glucose control was up to standard. Referring to the results of blood glucose, the bolus and basal rate of insulin pump before three meals were adjusted following the principles of 30 and 50, so as to keep the blood glucose stable. During treatment, attention should be paid to communication with patients, emphasizing the risk of diabetes and complications to the body, and correcting their bad habits. Without oral hypoglycemic agents, patients were guided to conduct reasonable diet and exercise to reduce the body's resistance to insulin. Insulin pump was removed after 2 weeks.

### 2.3. Ultrasonography

Color Doppler ultrasound machine was used. All subjects were placed in the supine or prone position with adequate exposure of the lower limbs. The probe was placed at the root of the thigh, along the course of the vessel, and the femoral artery, popliteal artery, posterior artery, anterior artery, and dorsalis pedis artery were scanned. The IMT of the vessel wall, the presence of plaques, the location of plaques, and their echo characteristics were observed and assessed by two-dimensional ultrasound images. The lumen filling condition was observed. The arterial spectrum was measured by spectral Doppler. The sampling volume was in the center of vascular cavity during sampling. The sampling volume was 1-3 mm. The scanning angle was adjusted so that the angle between acoustic beam and blood flow was ≤60°. Three to five consecutive spectra with consistent and clear morphology were recorded. The arterial analysis software was set in the instrument to measure the peak systolic velocity (PSV) and blood flow volume (BFV) of common femoral artery, popliteal artery, and dorsalis pedis artery. IMT was measured at the 1.5 cm posterior wall of the proximal segment of the common femoral artery bifurcation with reference to previous literature. Normal common femoral artery IMT < 1.0 mm and 1.0 mm ≤ IMT < 1.2 mm were considered thickened, and IMT ≥ 1.2 mm was plaque formation. The probe was placed at the carmine fossa, and IMT of the popliteal artery was measured at the posterior wall of the popliteal artery cross-section. IMT of the dorsalis pedis artery was measured in the transverse posterior wall 1 cm distal to the junction with the ankle joint. Each data was measured three times and averaged. All measurements were performed by the same physician on the same diagnostic ultrasound instrument.

### 2.4. Diagnostic Criteria for LEAD

Clinical symptoms: intermittent claudication, resting pain, etc.; physical examination: palpation of the dorsalis pedis artery, whether the pulse became weak or cannot be felt; relevant examinations: ankle-brachial index (ABI) ≤ 0.9; toe-brachial index (TBI) ≤ 0.7; lower limb artery color Doppler ultrasound revealed significant stenosis (single or multiple stenosis ≥ 50%) or occlusion; lower limb angiography revealed single or multiple severe stenosis (stenosis ≥ 50%) and/or occlusion of the iliac, femoral, carmine, and tibial and peroneal arteries of the lower leg. Based on typical symptoms and signs, the diagnosis can be confirmed if one of the examination items is positive [15]. The scoring criteria are shown in Table 1.

### 2.5. Observation Indicators

General conditions: the general data of all the patients were collected when the patient came for a follow-up visit, including gender, age, disease course, systolic pressure (SP), diastolic pressure (DP), and body mass index (BMI).

Collection of serological samples: patients admitted to the hospital were fasted for 10 h. About 3-5 mL of blood was collected from the vein the next morning, mixed well, and placed at room temperature. Observation Indicators include serum total cholesterol (TC), triglyceride (TG), low density lipoprotein cholesterol (LDL-C), and high density lipoprotein cholesterol (HDL-C), fasting plasma glucose (FPG), liver and kidney function, HbA1c, HCY.

### 2.6. Statistical Methods

SPSS16.0 was used for data analysis. Measurement data were expressed as mean ± standard deviation ($\overset{¯}{x}\pm s$) after normality test. The comparison of measurement data between the two groups was performed by two sample *t* test. The comparison of count data between the two groups was carried out by chi-square test. The correlation analysis of measurement data was performed by Pearson correlation test. *P* < 0.05 indicated that the difference was statistically significant.

## 3. Results

### 3.1. Basic Information of Patients in the Two Groups at First Visit

The average age of the control group was 45.42 ± 4.12 years old, the average course of disease was 10.11 ± 6.52 years, the average BMI level was 24.18 ± 1.34 kg/m^2^, and the average HCY was 12.01 ± 2.72 *μ*mol/L. The average age of the experimental group was 46.25 ± 3.28 years old, the average course of disease was 11.32 ± 5.39 years, the average BMI level was 24.93 ± 1.19 kg/m^2^, and the average HCY was 12.07 ± 2.74 *μ*mol/L. At the first visit, there was no significant difference in age, gender, BMI, and other general information and indicators between the control group and the experimental group (*P* > 0.05). The HbA1c level in the experimental group was higher at the first visit, which was 9.94 ± 1.74%; the HbA1c level in the control group was 8.02 ± 1.41%, and the difference between the two groups was statistically significant (*P* < 0.05). The LEAD scores of the two groups were compared after calculation. The experimental group had 1.01 ± 0.54 points, and the control group had 0.97 ± 0.55 points on average. There was no significant difference between the two groups (*P* > 0.05) (Table 2 and Figure 1).

### 3.2. Analysis of Ultrasonic Examination Results after Treatment

After two weeks of treatment, in the control group, 28 patients' lumen intima was smooth, 52 patients' lumen intima was not smooth but no plaque, and 131 patients' lumen intima was not smooth and there was plaque. In the experimental group, 69 patients' lumen intima was smooth, 101 patients' lumen intima was not smooth but no plaque, and 41 patients' lumen intima was not smooth and there was plaque. The difference between the two groups was statistically significant (*P* < 0.05) (Figure 2).

The comparison results of IMT, PSV, and BFV of the lower limb arteries in the two groups showed that in the experimental group, the IMT values of the common femoral artery, popliteal artery, and dorsalis pedis artery were 0.83 ± 0.03 mm, 0.62 ± 0.03 mm, and 0.41 ± 0.04 mm, respectively; the PSV values were 92.33 ± 19.01 cm/s, 61.14 ± 12.77 cm/s, and 42.26 ± 11.28 cm/s, respectively; BFV values were 290.77 ± 103.58 cm/s, 70.11 ± 36.33 cm/s, and 15.03 ± 8.95 cm/s, respectively; in the control group, the IMT values of common femoral artery, popliteal artery, and dorsalis pedis artery were 1.62 ± 0.54 mm, 1.23 ± 0.14 mm, and 0.78 ± 0.11 mm, respectively; the PSV values were 94.96 ± 19.47 cm/s, 62.87 ± 11.03 cm/s, and 44.12 ± 10.63 cm/s, respectively; the BFV values were 312.46 ± 109.87 cm/s, 77.92 ± 45.28 cm/s, and 14.88 ± 6.29 cm/s, respectively. Between the two groups, the arterial IMT values of the experimental group were lower than those of the control group, and the difference was statistically significant (*P* < 0.05). PSV and BFV values were lower than those of the control group, but the difference was not statistically significant (*P* > 0.05) (Figures 3–5).

### 3.3. Analysis of Serum Test Results after Treatment

After two weeks of treatment, the serum test results showed that there was no significant difference in the levels of TC, TG, and HDLC between the experimental group and the control group (*P* > 0.05). There was an obvious difference in LDL-C level between the experimental group (2.22 ± 0.46 mmol/L) and the control group (3.21 ± 0.62 mmol/L) (*P* < 0.05). The HCY level of the experimental group was 15.26 ± 2.64 *μ*mol/L; the HCY level of the control group was (17.83 ± 4.38 *μ*mol/L) (*P* < 0.05). The LEAD score of lower limb blood vessels in the experimental group was 5.51 ± 1.11; the LEAD score of lower limb blood vessels in the control group was 7.08 ± 2.73 (*P* < 0.05) (Figure 6).

### 3.4. Analysis of LEAD Score in Patients with Different Course of Disease

After two weeks of treatment, the results of LEAD scores of patients with different course of disease (CD) showed that when 1 < CD ≤ 5 years, the difference in LEAD scores between the two groups was small, without significant difference (*P* > 0.05); when 6 ≤ CD ≤ 10 years; the average score of patients in the experimental group was 5.39 ± 1.12 points, compared with 7.02 ± 2.73 points in the control group, the difference was statistically significant (*P* < 0.05); when CD > 10 years, the average score of patients in the experimental group was 6.01 ± 1.03 points, compared with 7.82 ± 2.39 points in the control group, the difference was statistically significant (*P* < 0.05) (Figure 7).

## 4. Discussion

Limb ischemia caused by diabetic LEAD is not only a factor causing the occurrence of diabetic foot but also an important cause of recurrent and prolonged diabetic foot ulcers [16]. LEAD in patients with DM has an insidious onset and usually atypical or even asymptomatic clinical symptoms, which makes DM patients and doctors often ignore the presence of LEAD, which makes it difficult to correctly diagnose and evaluate diabetic LEAD [17]. Therefore, it becomes particularly important for the early screening and assessment of LEAD in T2DM patients. 422 T2DM patients with LEAD were selected and evaluated the therapeutic effect by ultrasound images after insulin pump therapy. The results showed that there was no significant difference in age, gender, BMI, and other general data and indicators between the control group and the experimental group at initial diagnosis (*P* > 0.05); only in the comparison of HbA1c, the level of the experimental group was 9.94 ± 1.74%, which was significantly different from the level of the control group (8.02 ± 1.41%) (*P* < 0.05), indicating that the baseline data of the two groups were comparable.

After two weeks of treatment, the difference in the intimal condition between the two groups had statistical significance (*P* < 0.05); the IMT values of common femoral artery, popliteal artery, and dorsalis pedis artery in the experimental group were 0.83 ± 0.03 mm, 0.62 ± 0.03 mm, and 0.41 ± 0.04 mm, respectively; the IMT values of common femoral artery, popliteal artery, and dorsalis pedis artery in the control group were 1.62 ± 0.54 mm, 1.23 ± 0.14 mm, and 0.78 ± 0.11 mm, respectively; the IMT of artery in the experimental group was lower than that in the control group, and the difference had statistical significance (*P* < 0.05); although the PSV and BFV values were lower in the experimental group than those in the control group, the difference had no statistical significance (*P* > 0.05). Studies have shown that the reasons for no difference in hemodynamic changes of lower limb arteries may be (1) the endothelial cell function of lower limb arterial lesions in patients with T2DM is still intact, so that the hemodynamic changes are not obvious; (2) the early intima is rough and unsmooth, the intima-media thickening and plaque formation do not cause significant stenosis, so the hemodynamics may not change significantly. Later, the vascular lesions are gradually aggravated, causing significant stenosis, which will lead to hemodynamic abnormalities [18].

Studies indicated that the repair of islet function plays a regulatory role in HCY metabolism and improves oxidative stress in patients, thereby improving the long-term prognosis of patients [19]. It showed that after two weeks of treatment, HCY level was significantly lower in the experimental group, indicating that islet function was gradually repairing in patients. T2DM is closely related to severe glucose and lipid metabolism disorders and insulin resistance [20]. The LDL-C level in the experimental group was significantly different from that in the control group, which may be because insulin pump therapy improved the early metabolism of the patients. The average LEAD score of lower limb vessels in the experimental group was 5.51 ± 1.11 points, compared with the average 7.08 ± 2.73 points in the control group, the difference was statistically significant (*P* < 0.05), which indicated that the LEAD score was lower, and the blood lipid level control was more ideal in patients who applied insulin pump to lower blood glucose. The difference in LEAD scores between the two groups was not apparent until 6 years ≤ CD. It can be concluded that in T2DM patients treated with short-term insulin pump therapy, with the extension of the course of the disease, the occurrence and progression rates of LEAD were significantly slower than those in patients who did not use insulin pump for a short time.

## 5. Conclusion

After treatment with insulin pump in T2DM patients with LEAD, through the evaluation of ultrasound images, the results showed that ultrasound had important clinical value in the diagnosis of LEAD in patients with T2DM, and it could help clinicians master the shape of lower limb vessels and their hemodynamic status by assessing the intima-media of lower limb arteries and hemodynamic information; in patients treated with insulin pump, the HCY level was significantly reduced, the occurrence and progression rates of LEAD were significantly slowed down, which could effectively help T2DM patients to improve the LEAD status and had clinical application value. However, there are some limitations, the causal relationship between blood lipid levels and LEAD in T2DM still cannot be judged, and long-term, large-sample, multiregional prospective studies are needed to further explore its relationship and possible mechanism.

## Figures and Tables

**Figure 1:** Comparison of indicators at the first visit. ∗Compared with the control group, the difference was statistically significant, *P* < 0.05.

**Figure 2:** Comparison of vascular lumen intima of lower extremity. ∗Compared with the control group, *P* < 0.05.

**Figure 3:** Comparison of IMT of lower extremity arteries. ∗Compared with the control group, *P* < 0.05.

**Figure 4:** Comparison of PSV of lower extremity arteries.

**Figure 5:** Comparison of BFV of lower extremity arteries.

**Figure 6:** Comparison of serum test results after treatment. ∗Compared with the control group, *P* < 0.05.

**Figure 7:** Comparison of LEAD scores in patients with different CD. ∗Compared with the control group, *P* < 0.05.

**Table 1:** LEAD scoring.

Items	0	1	2	3	4
ABI	>0.9	0.8 < ABI ≤ 0.9	0.7 < ABI ≤ 0.8	0.6 < ABI ≤ 0.7	ABI ≤ 0.6
Intermittent claudication: the maximum distance walking at the speed of 70-80 m/min	Distance ≥400 m	300-399 m	200-299 m	100-199 m	<100 m or unable to walk
Pain	No pain	Postexercise pain	Occasional resting pain	Resting pain at night or frequent resting pain	Persistent resting pain
Sense of numbness	No numbness	Occasional numbness	Frequent numbness	Frequent numbness and other abnormal feelings	Persistent numbness
Whether ischemic ulcer exists or not	No open lesions	Superficial lesions	Wound depth reaching tendon, ligament, and joint	Deep ulcer, osteomyelitis, abscess sinus	Toe and/or partial foot gangrene

**Table 2:** General information of two groups of patients.

Grouping	Male (cases)	Female (cases)	Age/years old	Course of disease/years	BMI (kg/m^2^)	SP (mmHg)	DP (mmHg)
Control group	113	98	45.42 ± 4.12	10.11 ± 6.52	24.18 ± 1.34	132.11 ± 7.82	84.21 ± 8.31
Experimental group	124	87	46.25 ± 3.28	11.32 ± 5.39	24.93 ± 1.19	127.54 ± 7.33	81.36 ± 8.77

## Data Availability

The data used to support the findings of this study are available from the corresponding author upon request.

## References

[1] Cole J. B., Florez J. C. (2020). Genetics of diabetes mellitus and diabetes complications. *Nature Reviews Nephrology*.

[2] Lovic D., Piperidou A., Zografou I., Grassos H., Pittaras A., Manolis A. (2020). The growing epidemic of diabetes mellitus. *Current Vascular Pharmacology*.

[3] Papatheodorou K., Banach M., Bekiari E., Rizzo M., Edmonds M. (2018). Complications of diabetes 2017. *Journal of Diabetes Research*.

[4] Almourani R., Chinnakotla B., Patel R., Kurukulasuriya L. R., Sowers J. (2019). Diabetes and cardiovascular disease: an update. *Current Diabetes Reports*.

[5] Petrie J. R., Guzik T. J., Touyz R. M. (2018). Diabetes, hypertension, and cardiovascular disease: clinical insights and vascular mechanisms. *Canadian Journal of Cardiology*.

[6] Takahara M. (2021). Diabetes mellitus and lower extremity peripheral artery disease. *JMA Journal*.

[7] Bourron O. (2019). Artériopathie chez le patient diabétique [Lower limb arterial disease in patients with diabetes]. *La Revue du praticien*.

[8] Buso G., Aboyans V., Mazzolai L. (2019). Lower extremity artery disease in patients with type 2 diabetes. *European Journal of Preventive Cardiology*.

[9] Martinelli O., Alunno A., Drudi F. M., Malaj A., Irace L. (2021). Duplex ultrasound versus CT angiography for the treatment planning of lower-limb arterial disease. *Journal of Ultrasound*.

[10] Schicchi N., Fogante M., Oliva M. (2019). Radiation dose and image quality with new protocol in lower extremity computed tomography angiography. *La Radiologia Medica*.

[11] Cavallo A. U., Koktzoglou I., Edelman R. R. (2019). Noncontrast magnetic resonance angiography for the diagnosis of peripheral vascular disease. *Circulation. Cardiovascular Imaging*.

[12] Shabani Varaki E., Gargiulo G. D., Penkala S., Breen P. P. (2018). Peripheral vascular disease assessment in the lower limb: a review of current and emerging non-invasive diagnostic methods. *BioMedical Engineering OnLine*.

[13] Evans R. M., Wei Z. (2022). Interorgan crosstalk in pancreatic islet function and pathology. *FEBS Letters*.

[14] Freckmann G., Buck S., Waldenmaier D. (2021). Insulin pump therapy for patients with type 2 diabetes mellitus: evidence, current barriers, and new technologies. *Journal of Diabetes Science and Technology*.

[15] Poorthuis M. H. F., Morris D. R., de Borst G. J. (2021). Detection of asymptomatic carotid stenosis in patients with lower-extremity arterial disease: development and external validations of a risk score. *The British Journal of Surgery*.

[16] Choke E., Tang T. Y., Cheng S. C., Tay J. S. (2020). Treatment of lower limb ischaemia in patients with diabetes. *Diabetes Metab Res Rev*.

[17] Neagu C., Buzea A., Agache A., Georgescu D., Pătraşcu T. (2018). Surgical revascularization in chronic limb-threatening ischemia in diabetic patients. *Chirurgia*.

[18] Li X. Y., Jiao Y., Zhou X. L. (2018). Effect of standardized treatment on reactivity of toe microcirculation in patients with type 2 diabetes mellitus. *Zhonghua Yi Xue Za Zhi*.

[19] Yuan X., Ding S., Zhou L., Wen S., Du A., Diao J. (2021). Association between plasma homocysteine levels and pancreatic islet beta-cell function in the patients with type 2 diabetes mellitus: a cross-sectional study from China. *Annals of Palliative Medicine*.

[20] Zhang Z., Wang J., Wang H. (2018). Correlation of blood glucose, serum chemerin and insulin resistance with NAFLD in patients with type 2 diabetes mellitus. *Experimental and Therapeutic Medicine*.

